# Survival as a Function of Nonsteroidal Anti-inflammatory Drug Use in Patients with Glioblastoma

**DOI:** 10.7759/cureus.3277

**Published:** 2018-09-10

**Authors:** Ryan P Bruhns, Whitney S James, Mohammad Torabi, Mark Borgstrom, Adam Roussas, Michael Lemole

**Affiliations:** 1 Surgery, Banner University Medical Center, Tucson, USA; 2 Neurological Surgery, Banner University Medical Center, Tucson, USA; 3 Research and Computing, University of Arizona, Tucson, USA; 4 Surgery, Banner University Medical, Tucson, USA; 5 University of Arizona

**Keywords:** stupp regimen, survival, tumor, non-steroidal anti-inflammatory drugs (nsaid), brain

## Abstract

Background

Findings of both case control and in vitro investigations suggest that non-steroidal anti-inflammatory drugs (NSAIDs) may play a beneficial role in the occurrence, growth, and subsistence of glioblastoma multiforme (GBM) brain tumor in humans.

Objective

In the present retrospective cohort study, we assessed the impact of NSAID use on survival in patients diagnosed with and treated for GBM brain tumors.

Methods

The impact of NSAID use and six other potential prognostic indicators of survival were assessed in 71 patients treated for GBM brain tumors from February 2011 to June 2016. Survival analysis and cross-tabulation analyses were performed to examine the potential relationship between NSAID use and occurrence of intracranial hemorrhage over the course of treatment for GBM.

Results

Kaplan-Meier analysis revealed no significant difference in survival between patients with and without NSAID use (p = 0.75; 95% CI: 10.12, 18.13). Multiple Cox regression analysis identified only treatment with chemotherapy as imposing any statistically significant effect on survival (Hazard Ratio (HR) = 3.31; p < 0.001; 95% CI: 1.80, 6.07). Cross-tabulation revealed no significant effect of NSAID use on occurrence of hemorrhage during treatment, X^2^ (2, N = 71) = 0.65, p_2-Sided_ = 0.42, (Fisher’s Exact Test: p2-sided = 0.56, p1-sided = 0.31).

Conclusion

These results suggest that history of NSAID use is not a determinant of survival in GBM patients. More rigorous, prospective investigations of the effect of NSAID use on tumor progression are necessary before the utility of this family of drugs in the treatment of GBM can be adequately appraised.

## Introduction

Glioblastoma multiforme (GBM) is the most aggressive and commonly occurring primary intracranial tumor, conferring a median survival of 10–14 months following multi-modal treatment [1]. Despite its recalcitrance in the face of the currently dominant therapeutic model, i.e., surgical resection, radiation therapy, and chemotherapy with temozolomide (TMZ) [2, 3], recent investigations have demonstrated responsiveness of GBM cells to treatment with non-steroidal anti-inflammatory drugs (NSAIDs). Sareddy et al. (2012) described the dose-dependent, anti-proliferative, and pro-apoptotic effects of the non-reversible COX-2 inhibitor, celecoxib, in GBM cell lines, demonstrating its potential inhibitory roll in the NF-κB pathway [4]. The upregulation and activation of this pathway is observed in GBM and implicated as a significant driver of gliomagenesis and its resistance to treatment with O6-alkylating agents, in particular [5]. Recently, celecoxib was found to exert similar antiproliferative effects and increase the radiosensitivity of certain GBM cell lines under normoxic and hypoxic conditions [6].

Inhibitors of COX-1 have been found to serve antagonistic roles in glioma cell survival and proliferation. Bernardi et al. (2013) described reduced viability of glioma cells through induced apoptosis, cell-cycle arrest, and increased differentiation following targeted administration of indomethacin-loaded lipid-core nanocapsules to C6 and U138-MG glioma cell lines [7]. Furthermore, synergistic sensitization of glioblastoma cells to TMZ was observed after administration of aspirin-loaded poly-lactic-co-glycolic acid (PLGA) microspheres to LN229 and U87 glioma cell lines [8]. Of note, arachidonic acid metabolites, particularly those of the cyclooxygenase pathway, have been implicated in the growth and subsistence of human and rat brain tumors in vitro and in vivo, respectively [9]. Pathways in addition to those of COX-1 or -2 have been identified [10, 11], suggesting a potentially wide variety of effects of NSAIDs on glioma cell lines. Examples include the upregulation of 15-hydroxyprostaglandin dehydrogenase (15-PGDH, a key inactivator of prostaglandins) and the cell cycle regulator p21 in GBM cell lines treated with dissolved Diclofenac sodium and meloxicam sodium [10].

The investigated in vitro effects of NSAIDs on GBM cell lines have yet to be comprehensively translated clinically. The association between chronic NSAID use and risk of GBM in humans was investigated by Sivak-Sears et al. (2004) through a case-control study including 236 GBM cases and 401 unaffected, age-, gender-, and ethnicity-matched controls [12]. The first study of its kind, the authors concluded that use of at least 600 pills of aspirin, ibuprofen, naproxen, and/or any other NSAIDs, and acetaminophen during the 10-year pre-diagnostic or pre-interview period was significantly inversely associated with the occurrence of histologically-confirmed GBM. The inverse correlation was noted to persist even following the exclusion of data for NSAID use initiated two years prior to diagnosis (a measure to control for increased use between the period of tumor induction and onset of clinical symptoms) [12]. There is currently a paucity of clinical research investigating the roll of NSAID use in GBM tumor progression. In the present retrospective cohort study, we assessed the impact of NSAID use on survival in patients diagnosed with and treated for GBM brain tumors.

## Materials and methods

After obtaining Institutional Review Board approval, a retrospective chart review of neurosurgical patients at Banner University Medical Center in Tucson, Arizona was conducted to identify all patients with new or pre-existing diagnoses of GBM presenting from February 2011 to June 2016. Patient consent was neither required nor sought due to the retrospective nature of this investigation, in addition to the de-identification of all information pertaining to study participants. Electronic medical records (EMR) of patients with GBM were individually reviewed and the following information: age, sex, date of GBM diagnosis, date of death (if applicable), whether the patient underwent gross total resection (GTR) of the tumor, whether the patient underwent chemotherapy with temozolomide (with or without treatment with bevacizumab), whether the patient received radiation therapy, tumor location, NSAID use, history of other cancers, and whether the patient suffered any intracranial hemorrhage over the course of their tumor treatment. Tumor locations were coded into three distinct groups: (1) superficial/cortical tumors, (2) basal ganglia, brain stem, thalamic, or cerebellar tumors, and (3) bilateral/interhemispheric tumors. Patients whose electronic record did not indicate biopsy-confirmed GBM were excluded from the study.

Survival from time of diagnosis was calculated as the difference (in months) of the date of death and the date of diagnosis. A subset of the considered patient population lacked explicitly documented dates of death, but were nevertheless noted in their electronic records to be deceased or to have been referred to a palliative care facility in poor condition. For these patients, the last documented date of correspondence was substituted for date of death. Patients whose EMR indicated a stable condition upon their most recent evaluation were assumed to be alive. Determinations of NSAID use were based on home medication lists recorded upon initial presentation, with usage defined as having been taking any oral NSAID either daily or as needed up to the date of initial presentation. Patients who were prescribed NSAIDS after the initial diagnosis of GBM were not considered for inclusion in the study. The electronic medical records of 76 patients diagnosed with GBM were reviewed. Five were excluded from the study for absence of biopsy confirmation, ambiguity of the pathology report, or other missing values. Ten patients were alive as of June 2016.

Survival analyses were performed on 71 patients using the Mantel-Cox log rank test for the comparison of Kaplan-Meier survival curves and the Cox proportional hazards model. A cross tabulation was also performed to examine the potential relationship between NSAID use and occurrence of intracranial hemorrhage over the course of GBM treatment. Between-group comparisons were examined using Fisher’s exact and Pearson’s Chi-Squared tests. These analyses were performed using SPSS version 24.0 for Windows (IBM, Armonk, NY).

## Results

Patient demographic and clinical course characteristics

In total, 71 patient cases (45 (63.4%) male; median age = 59) were reviewed for analysis. Of these, 84.5% of patients underwent GTR, 73.2% received chemotherapy, 74.6% received radiation therapy, 70.4% received both chemotherapy and radiation, 12.7% had a history of cancer other than GBM, 26.8% experienced intracranial hemorrhage over the course of tumor treatment, and 28.2% were using NSAIDs prior to undergoing treatment related to their GBM brain tumor. Of patients with recorded, prior NSAID use, 95% underwent GTR, 65% received chemotherapy, 75% received radiation therapy, and 60% received all three interventions. The distribution of tumor location at the time of diagnosis was largely skewed toward neoplasms of superficial/cortical origin (80.3%), followed by tumors originating in the basal ganglia, thalamus, brain stem, or cerebellum (14.1 %) and those presenting bilaterally (5.6%) (Table 1).

**Table 1:** Patient demographics and clinical characteristics. GBM: Glioblastoma multiforme; NSAID: Non-steroidal anti-inflammatory drug.

Demographics of Patient Sample	Frequency (%)
Age (Median)	59
Females	26 (36.6)
Males	45 (63.4)
NSAID Use	20 (28.2)
Surgical Resection of Tumor	60 (84.5)
Chemotherapy	52 (73.2)
Radiation	53 (74.6)
Chemotherapy and Radiation	50 (70.4)
Tumor Located Superficially in Cortex	57 (80.3)
Tumor Located in Basal Ganglia, Thalamus, Brain Stem, or Cerebellum	10 (14.1)
Tumor is Interhemispheric or Bilateral	4 (5.6)
History of Cancer Other than GBM	9 (12.7)
Intracranial Hemorrhage During GBM Treatment	19 (26.8)

Analysis of survival

The overall post-diagnosis survival of sampled patients ranged from 0 to 71 months (M = 11.98 months, SD = 13.97 months). Kaplan-Meier analysis revealed no significant difference in survival between patients with and without NSAID use (p = 0.75) (Figure 1). Multiple regression analysis identified only treatment with chemotherapy as imposing any statistically significant effect on survival (p < 0.001) (Figure 2). A single Cox regression analysis also demonstrated a lack of statistically significant effect of NSAID use on survival (p = 0.76; 95% CI: 0.62–1.95) (Figure 3).

**Figure 1:** Kaplan-Meier survival curve comparing usage and non-usage of NSAIDs. A relative increase in percent survival in the curve of NSAID users over that of non-NSAID users can be appreciated from approximately 10 months to 40 months, however this finding is not statistically significant. NSAID: Non-steroidal anti-inflammatory drug

**Figure 2:** Cox regression depicting the results of the combined proportional hazards analysis. Chemotherapy is an independent prognostic indicator of survival (p < 0.001).

**Figure 3:** Cox regression analysis. Demonstrates a null effect of NSAID use on survival probability in patients diagnosed with GBM (p = 0.76). NSAID: Non-steroidal anti-inflammatory drug; GBM: Glioblastoma multiforme.

Cross tabulation

A comparison of the relationship between NSAID use and occurrence of intracranial hemorrhage over the course of treatment (Figure 4) did not yield a significant negative correlation, suggesting no significant effect of NSAIDs on intracranial hemorrhage (p = 0.42).

**Figure 4:** Occurrence of intracranial hemorrhage in patients with and without NSAID use during the course of GBM treatment. There is a modest, though not significant, negative correlation between the condition of NSAID use and the occurrence of hemorrhage, X^2 ^(2, N = 71) = 0.65, p2-Sided = 0.42 (Fisher’s Exact Test: p_2-sided_ = 0.56, p1-sided = 0.31). GBM: Glioblastoma multiforme; NSAID: Non-steroidal anti-inflammatory drug.

## Discussion

The results of the present study do not support the role of history of NSAID use as an important determinant of survival in patients diagnosed with and treated for GBM brain tumor. A weak, positive effect of NSAID use on percent survival was noted following Kaplan-Meier analysis (Figure 1) from approximately 10 to 40 months post-diagnosis. This effect, though not statistically significant (p = 0.75 (Mantel-Cox)), warrants further investigation, as it could be due only to a correlation of NSAID use with other independent variables in the model. Corroborating this, the results of the independent Cox proportional hazards model examining NSAID use alone on survival probability post-GBM diagnosis (Figure 3) indicate a lack of statistical significance, even when examined separately from the more influential (and thereby masking) effect of treatment with chemotherapy, X^2^ (2, N = 71) = 0.095, p = 0.76.

Not surprisingly, the results of the multiple regression analysis (Cox regression) implicate treatment with chemotherapy, a common adjuvant to GTR and radiotherapy, as the major prognostic indicator in patients with GBM. The effect measure indicating this, the ‘Exp(B)’ value (Exp(B)Chemotherapy = 3.31), can be interpreted as the odds ratio, or hazard ratio, comparing the probability of survival in an individual treated with chemotherapy to an individual who does not undergo chemotherapy. That is, in this sample, the odds of survival for an individual treated with chemotherapy were 3.31 times those of an individual not treated with chemotherapy. However, limitations exist in this investigation’s ability to conclude that this effect is due uniquely to temozolomide treatment, for example, and not to combined chemotherapeutic, radiotherapeutic, and surgical measures as these treatments are generally offered together. This limitation exists chiefly because of an inability to cleanly separate prognostic factors when they are examined using a proportional hazards model. Still, this finding is in agreement with previous investigations of GBM patients, which name concomitant or adjuvant chemotherapy, particularly with temozolomide, as significantly improving survival outcomes in GBM patients, especially those whose tumor cells express MGMT [13]. Conclusions suggesting improved or diminished effects in elderly patients, however, are mixed [14]. Results of the cross tabulation analysis demonstrate a similarly null effect of NSAID use on the occurrence of intracranial hemorrhage over the course of treatment for GBM. It is possible that this effect would be more pronounced and, thus, reach statistical significance if a larger sample of patients were to be analyzed; however, because the manner by which intracranial hemorrhage (whether pre-, intra-, or post-operative) and other variables are reported is remarkably inconsistent in terms of the location and timeliness of electronic documentation, it remains difficult to capture all events in question.

These data build on those of Sivak-Sears et al. (2004), which demonstrate an inverse correlation between chronic NSAID use and GBM status, both self-reported, i.e., data were obtained verbally from in-person interviews with patients, proxies, and controls after they were mailed packets containing information on topics relevant to the investigation [12]. As discussed by the authors of the study, this method of data collection was a possible limitation to the reliability of results obtained. As such, the findings warranted corroboration by further study of GBM development or progression, taking into consideration individual NSAID usage. The present study, through the incorporation of biopsy-confirmed GBM status and physician-collected medication information, may be viewed as exhibiting improved reliability of data collected for both independent and dependent factors.

Apart from the general, established limitations of studies incorporating retrospective chart reviews, other limitations of this investigation include the fact that survival outcomes were not stratified based upon grade or stage of the tumor, age of the patient at presentation, molecular markers (e.g., MGMT expression and/or IDH1 mutation status), or tumor size. All of these constitute established prognostic factors of survival in GBM patients that may have masked the effect of lesser independent variables such as NSAID use in the models used by the aforementioned survival analyses [15,16]. Conversely, NSAID use, as described above, may simply be correlated with other factors examined by the model, limiting the interpretation of positive effects on survival percentage and probability. For example, a patient who takes NSAIDs chronically may be more likely to accept chemotherapy as a treatment, with the survival benefit to follow being due to the chemotherapy regime rather than to NSAID use. To control for chemotherapy in this investigation would mean considering only the 19 patients who did not receive it, of whom only seven were using NSAIDs. Also of note, this retrospective investigation does not account for those patients whose GBM diagnoses came early or late relative to tumor induction, introducing a potential lead-time bias. However, being that no effect was observed for the NSAID condition following initial analyses, calculation of back-end survival to correct for lead-time was deemed unnecessary. Finally, the retrospective nature of this study did not permit specification of NSAID use duration or frequency prior to GBM diagnosis. It is possible that some patients were taking NSAIDs for one month prior to GBM diagnosis while others were taking them for years prior to diagnosis, and these discrepancies in duration of NSAID use could have weakened possible correlations in survival.

The present study represents an exploratory effort to determine what effect, if any, NSAID use has on the progression of a malignancy that carries a historically dismal prognosis. Taking into consideration the above points, it is clear that attempts to answer this question using retrospective analyses to examine small hospital samples come with numerous caveats. For this reason, further prospective investigation incorporating larger samples is necessary to more firmly establish or refute a connection between NSAIDs and GBM induction, progression, and survival following diagnosis. This would seem a worthy pursuit not only on the basis of the equivocality of findings obtained to date, but also on that of the sheer potential of an inexpensive and accessible addition to the GBM treatment armamentarium.

## Conclusions

The present retrospective chart review examined the role of NSAID use, as well as six other potential prognostic indicators of survival time in 71 patients with GBM brain tumor using two distinct analyses of survival. Of the seven independent factors examined, only treatment with chemotherapy was found to have a positive effect on survival post-diagnosis. Moreover, survival analysis did not identify a significant effect of NSAID use or any of the other five factors examined on survival outcomes in patients with biopsy-confirmed GBM brain tumor. However, 84.5% and 74.6% of the sample received surgical and radiation therapies, respectively, making unclear the individual contributions of each with respect to the dominant prognostic indicator: treatment with chemotherapy. These findings suggest a need for further, more rigorous, prospective investigation of the effect of NSAID use on tumor progression before the utility of this family of drugs in the treatment of GBM can be adequately appraised.
